# Effects of C5a and Receptor CD88 on Glutamate and N-Methyl-D-Aspartic Acid Receptor Expression in the Mouse Model of Optic Neuromyelitis

**DOI:** 10.1155/2022/4997393

**Published:** 2022-04-25

**Authors:** Ling Li, Jiangwei Tang, Hongxin Wang, Jiamei Liu, Lina Zhou

**Affiliations:** Department of Neurology, Tianjin No.4 Central Hospital, Tianjin 300000, China

## Abstract

**Objective:**

To analyze the role of C5a, C5a receptor (CD88), glutamic acid, and N-methyl-D-aspartic acid receptors (NMDAR1 and NMDAR2B) in the onset of neuromyelitis optica (NMO) disease in mice.

**Method:**

To select C57BL/6 wild-type (WT) mice and C5a receptor gene knockout (C5aR-/-) mice, use NMO-IgG and hemolytic complement to intervene in spinal cord tissue sections and optic nerves to establish an NMO model *in vitro*. The experiment was carried out with five groups (control group, WT group, C5aR-/- group, C5a group, and C5a+C5aRA group), with six mice in each group. The differences of American spinal cord injury (ASIA) motor scores were compared among all groups. The expressions of aquaporin (AQP4), glial fibrillary acidic protein (GFAP), NMDAR1, and NMDAR2B in spinal cord and optic nerve tissues were detected. The difference of glutamic acid (Glu) concentrations in culture solutions of the spinal cord and optic nerves was compared.

**Result:**

The ASIA motor score of the control group was significantly lower than that of the other four groups. The C5a-/- group was significantly higher than the WT group. The C5a+C5aRA group was significantly higher than the C5a group in terms of ASIA motor score. In the control group, AQP4 and GFAP showed expression loss. The C5aR-/- group's loss rate was significantly higher than that of the WT group. The loss rate of the C5a+C5aRA group was significantly higher than that of the C5a group. In the control group, the protein expressions of NMDAR1 and NMDAR2B were significantly lower than that of the other four groups. The C5aR-/- group was significantly higher than the WT group. The C5a+C5aRA group was significantly higher than the C5a group in protein expression. In the control group, the concentration of Glu in the C5aR-/- group was significantly higher than that in the WT group, and the C5a group was significantly lower than the C5a+C5aRA group.

**Conclusion:**

The deletion of the C5a receptor promotes NMDAR activity, which affects the toxic excitatory effect of NMDAR in NMO and regulates the neurotoxic effect of glutamic acid, thus participating in the pathogenesis of NMO.

## 1. Introduction

Neuromyelitis optica (NMO) is a common inflammatory demyelinating disease in the central nervous system, which is usually related to vision. It also may cause pain and discomfort on one or both sides of the eyeball. The main pathological changes of patients with NMO are extensive axon loss and demyelination of myelin sheath [1, 2]. Glutamate (Glu) is a critical neurotransmitter in the central nervous system that plays a vital role in cell membrane potential homeostasis and cell microenvironment homeostasis [3]. The research suggested that pathologically speaking, the abnormal release of Glu or metastasis disorder can lead to abnormal accumulation of Glu in the synaptic cleft. As a result, the related receptors on the membrane would be stimulated to mediate the abnormal influx of sodium and calcium ions, causing the change of membrane potential and damaging cell microenvironment homeostasis, which eventually leads to cell apoptosis. It is closely related to cell energy metabolism, mitochondrial function, and antioxidant function [4, 5]. N-Methyl-D-aspartic acid receptor (NMDAR) is a Glu receptor, which is often closely related to the occurrence of central neuroinflammatory demyelinating diseases such as multiple sclerosis and autoimmune encephalomyelitis. NMDAR2B plays an important role in glutamate-induced excitatory nerve injury, and its increased activity can induce excitatory nerve injury in oligodendrocytes, which mediates demyelination of the central nervous system and optic nerve [6, 7]. Thus, its role in inflammatory demyelinating disease NMO has come into focus. Anaphylatoxin C5 is an essential component of the complement system, and its activM, lated cleavage fragment C5a is an important inflammatory mediator. The C5a/C5aR-related signaling pathway plays a significant role in the regulation of inflammatory response. A previous study has demonstrated that C5a may attract phagocytes with specific receptors, including microglia and astrocytes, to aggregate to the inflammatory site and expand the local inflammatory response, thus forming a neurotoxic inflammatory environment leading to neuronal dysfunction [8, 9]. At present, the interaction between C5a, NMDAR, and Glu is still unclear. In this study, the role of C5a and its receptor C5aR in NMO was explored by constructing an *in vitro* neuromyelitis optic model. Also, the effects of C5a on the expression levels of NMDAR and Glu were investigated to explore the possible pathogenic mechanism of NMO.

## 2. Materials and Methods

### 2.1. Experimental Animals

The experiment was carried out by selecting specific pathogen-free (SPF) C57BL/6 wild-type (WT) mice and C5a receptor gene knockout (C5aR-/-) mice aged from 7 to 14 days old. All the mice were kept in an animal house with humidity at (52 ± 2)% and temperature at (25 ± 3)°C. These animals were fed on a standard 12 h light/dark cycle in a free access environment for one week. The experimental animals were all from Guangdong Animal Experiment Center and approved by our hospital's ethics committee.

### 2.2. Main Reagents

The main reagents are as follows: fetal bovine serum (FBS) (GIBCO, USA); mixed normal complement serum (Innovative Research, USA); rabbit anti-mouse NMDAR1 monoclonal antibody, rabbit anti-mouse NMDAR1 polyclonal antibody, rabbit anti-mouse AQP4 polyclonal antibody, and sheep anti-mouse GFAP polyclonal antibody (Abcam, USA); BCA Protein Quantitation Kit (Invitrogen, USA); Glu detection kit (Beyotime Biotechnology, China); and recombinant human C5a and C5aR blocking agent (Fmoc Boc, Shanghai, China).

### 2.3. Model Preparation of NMO and Grouping

C57BL/6 WT mice and C5aR-/- mice aged 7 to 14 days were selected. The mice were killed by decapitation. Spinal cord tissue was isolated from spinal diseases of mice. The spinal cord tissue was placed on an agar block to prepare continuous sections with a thickness of about 300 *μ*m. Later, spinal cord tissue sections were placed on a 30 mm 4 *μ*m transwell membrane for routine culture, and the culture solution was replaced every three days. On the seventh day, the culture solution of the WT and C5aR-/- groups was replaced by a complete culture solution containing 300 *μ*g/mL NMO-IgG+10% normal complement serum. At the same time, in the WT group, no NMO-IgG+10% normal complement serum was set as the blank control group. Recombinant human C5a (50 nM) and recombinant human C5a (50 nM)+C5aR blocking agent (0.45 *μ*g/mL) were added to the WT group for 24 h. They were denoted as the C5a group and the C5a+C5aRA group, respectively. There were six mice in each group. Sections of all groups were cultured for three days, and an NMO spinal cord section model was prepared.

C57BL/6 WT mice aged six to eight weeks and C5aR-/- mice were selected. The mice were killed by decapitation. The mouse optic nerve was isolated and prepared into 300 *μ*m continuous sections and placed on a 30 mm 4 *μ*m transwell membrane for routine culture. Twenty-four hours later, the culture solution was supplemented with 300 *μ*g/mL NMO-IgG+10% normal complement serum, which was recorded as the WT group and the C5aR-/- group. At the same time, in the WT group, no NMO-IgG+10% normal complement serum was set as the blank control group. Recombinant human C5a (50 nM) and recombinant human C5a (50 nM)+C5aR blocking agent (0.45 *μ*g/mL) were added to the WT group for 24 h. They were denoted as the C5a group and the C5aRA group, respectively, with six mice in each group. Sections of all groups were cultured for 24 h, and an NMO optic nerve section model was prepared. All sections were fixed with 4% paraformaldehyde for reserve, and culture solution was collected for glutamate concentration detection.

### 2.4. Immunofluorescence Method Was Conducted to Detect AQP4 and GFAP Expressions

Spinal cord tissue and optic nerve tissue sections of each group were fixed with 4% polymethanol. Later, they were baked in the oven for 30 minutes. After the xylene was washed out with gradient alcohol (xylene dewaxing) and after phosphate buffer saline (PBS) washing, high-pressure antigen repair was conducted, then sealed with hydrogen peroxide; 10% normal goat serum was used to infiltrate the tissue. Optic nerve tissue was sealed at room temperature for 10 minutes, and spinal cord tissue was sealed with PBS containing 1% bovine serum protein and 0.3% Triton X-100 for an hour. After washing out, AQP4 and GFAP antibodies were added and incubated for the night at 4°C. The next day, the tissue sections were taken out and rewarmed to room temperature. After washing, a fluorescent secondary antibody was added, and samples were incubated at 37°C for an hour. After washing out again, fluorescence attenuation sealant was added to seal the sections.

Under the high-power field of an inverted microscope (×40), the expressions of AQP4 and GFAP in spinal cord tissue sections were observed. Under a high-power field (×200), the expression of AQP4 and GFAP in optic nerve tissue sections was observed.

### 2.5. NMO ASIA Motor Score

The integral optical density (IOD) and positive total area (area) of each field were measured utilizing Image-Pro Plus 6.0 software. ASIA motor score was carried out according to the expression of AQP4 and GFAP in each tissue section. A score of zero means that AQP4 and GFAP staining and sections were intact. A score of one means that AQP4 staining was weak; the astrocytes were swollen; the sections were intact. A score of two means that AQP4 and GFAP in more than one area of the section were completely lost and the area that was lost was less than 30% of the whole section. A score of three means that there were more than two areas of AQP4 and GFAP lost in the section and the area that was lost accounted for 30–80% of the whole section. A score of four means that the AQP4 and GFAP were lost in the sections and the area that was lost was greater than 80% of the whole section.

### 2.6. Glutamate Concentration Determined Based on Colorimetry

A Glu detection kit was adopted to detect Glu concentrations of culture solution. A sample was added to a 96-orifice plate, 25 *μ*L distilled water and 75 *μ*L reagent mixture were added to the blank well, and 25 *μ*L 200 *μ*mol/L glutamate standard application solution and 75 *μ*L reagent mixture were added to the standard well. 25 *μ*L supernatant and 75 *μ*L reagent mixture were added to the test orifice plate. The sample was carefully beaten and mixed with a pipette tip. The 96-orifice plate was placed on the enzyme plate analyzer, and the absorbance of each well was measured at 340 nm and recorded as the value A1. Later, 1 *μ*L reagent 5 was added to each well of the 96-orifice plate and incubated at 37°C for 40 minutes. Then, the 96-orifice plate was placed on the enzyme plate analyzer, and the absorbance of each well was measured at 340 nm, which was recorded as an A2 value. Glutamate concentration in culture solution was calculated according to the formula: Concentration of Glu (*μ*mol/L) = [(Measured A2 value − Measured A1 value) − (Blank A2 value − Blank A1 value)]/[(Standard A2 value − Standard A1 value) − (Blank A2 value − Blank A1 value)] × standard product concentration (200 *μ*mol/L) × dilution ratio before the sample test.

### 2.7. Western Blot Experiment Performed to Detect Protein Expressions of NMDAR1 and NMDAR2B

About 100 mg of tissues of each group was taken. Ophthalmic scissors were used to cut the tissue into tiny pieces. Later, the phenylmethylsulphonyl fluoride membrane protein extraction reagent was added, carefully beaten, mixed with a pipette head, and placed on ice to split decomposition for 15 minutes. The tissue suspension was collected into the homogenizer and observed under a microscope. If 70–80% of the cells had no perinuclear halo or intact cell morphology, it indicated that the homogenate was sufficient and the cells were fully cracked, which could be used for the next experiment. The tissue homogenate was transferred to the centrifuge tube and was centrifuged at 800 r/min at 4°C for 10 minutes; then, the supernatant was absorbed. It was then centrifuged at 12,000 r/min at 4°C for 20 minutes, and the supernatant remained at 30–50 *μ*L. The liquid supernatant was then abandoned. After centrifugation at 12,000 r/min at 4°C for 30 s, an appropriate amount of membrane protein extraction reagent B was added to resuspend the precipitation. It then underwent ice incubation for 10 minutes at 4°C, centrifuged at 12,000 r/min for 5 minutes, and the supernatant was collected and stored at -80°C for standby. The extracted protein was quantified using the BCA (bicinchoninic acid) Protein Quantitation Kit, and the protein content was calculated according to the standard curve. The extracted protein(s) of each group was loaded with 30–60 *μ*g of the same amount of protein, boiled, and denatured, and 10% sodium dodecyl sulphate–polyacrylamide gel electrophoresis SDS-PAGE gel electrophoresis was performed. After completing electrodeposited coating, the cells were transferred to a polyvinylidene fluoride membrane with a semidry blotter and then closed with 5% skim milk for an hour, followed by dilution of the primary antibody with 1% skim milk and incubation at 4°C overnight. The next day, the primary antibody was eluted with Tris-buffered saline+Tween, the secondary antibody was incubated at 37°C for an hour and developed with a chemical luminescent agent. Protein expressions of samples in NMDAR1 and NMDAR2B in each group were observed.

### 2.8. Statistical Treatment

SPSS 20.0 statistical software was adopted for data processing. Measurement data conforming to the normal distribution was expressed as mean ± standard deviation. If the data were conforming to the normal distribution and if the variance is homogenous, two independent sample *t*-tests would be used. If the variances are not uniform, the approximate *t*-test can be used. *P* < 0.05 means the difference is of statistical significance.

## 3. Result

### 3.1. Comparison of ASIA Motor Scores in Each Group

Compared with the control group, the spinal ASIA motor scores in the WT group and C5aR-/-, C5a, and C5a+C5aRA groups were significantly higher (*P* < 0.05). There was no significant difference in spinal cord injury scores between the C5aR and the WT groups (*P* > 0.05). The level of spinal cord injury in the C5a+C5aRA group was significantly higher than that in the C5a group (*P* < 0.05). There was no significant difference in spinal cord injury scores between the C5aR-/- group and the C5a+C5aRA group (*P* > 0.05), as shown in Figure 1.

### 3.2. Comparison of the Expression of AQP4 and GFAP in Spinal Cord Tissue Samples of Each Group

There was no deletion of AQP4 and GFAP staining in the spinal cord tissue of the control group. The absence of AQP4 and GFAP staining was detected in the WT group and C5aR-/-, C5a, and C5a+C5aRA groups. Also, the loss rate of AQP4 and GFAP staining in the C5aR-/- group was significantly higher than that in the WT group (*P* < 0.05). The loss rate of AQP4 and GFAP staining in the C5a+C5aRA group was significantly higher than that in the C5a group (*P* < 0.05), as shown in Figure 2.

### 3.3. Comparison of the Expression of AQP4 and GFAP in Optic Nerve Tissue Samples of Each Group

In the nerve tissue sample of the control group, there was no deletion of AQP4 and GFAP staining in the spinal cord tissue. The absence of AQP4 and GFAP staining was detected in the WT group and C5aR-/-, C5a, and C5a+C5aRA groups. Also, the loss rate of AQP4 and GFAP staining in the C5aR-/- group was significantly higher than that in the WT group (*P* < 0.05). The loss rate of AQP4 and GFAP staining in the C5a+C5aRA group was significantly higher than that in the C5a group (*P* < 0.05), as shown in Figure 3.

### 3.4. Comparison of Protein Expressions of Spinal Cord Tissue Samples in NMDAR1 and NMDAR2B in Each Group

According to the western blot experimental results, the protein levels of NMDAR1 and NMDAR2B in spinal cord tissue of the WT, C5aR-/-, C5a, and C5a+C5aRA groups were significantly higher than those of the control group (*P* < 0.05). The protein levels of NMDAR1 and NMDAR2B in the C5aR-/- group were significantly higher than those in the WT group (*P* < 0.05). The protein expressions of NMDAR1 and NMDAR2B in the C5a+C5aRA group were significantly higher than those in the C5a group (*P* < 0.05), as shown in Figure 4.

### 3.5. Comparison of the Protein Expression of NMDAR1 and NMDAR2B in Optic Nerve Tissue Samples of Each Group

Compared with the control group, the protein expression levels of NMDAR1 and NMDAR2B in the WT, C5aR-/-, C5a, and C5a+C5aRA groups were significantly higher (*P* < 0.05). The protein expression levels of NMDAR1 and NMDAR2B in the C5aR-/- group were significantly higher than those in the WT group (*P* < 0.05). The protein expression levels of NMDAR1 and NMDAR2B in the C5a group were lower than those in the C5a+C5aRA group (*P* < 0.05), as shown in Figure 5.

### 3.6. Comparison of Glu Concentration in Culture Solution of Spinal Cord Tissue of Each Group

Compared with the control group, the concentration of Glu in spinal cord tissue's culture solution of the WT, C5aR-/-, C5a, and C5a+C5aRA groups was significantly higher (*P* < 0.05). Glu concentration in the C5aR-/- group was significantly higher than that in the WT group (*P* < 0.05). Glu concentration in the C5a+C5aRA group was significantly higher than that in the C5a group (*P* < 0.05), as shown in Figure 6.

### 3.7. Comparison of Glu Concentration in Culture Solution of Optic Nerve Tissue of Each Group

The concentration of Glu in the culture solution of optic nerve tissue in the WT, C5aR-/-, C5a, and C5a+C5aRA groups was significantly higher than that in the control group (*P* < 0.05). Glu concentration in tissue culture solution in the C5aR-/- group was significantly higher than that in the WT group (*P* < 0.05). Glu concentration in the C5a group was significantly higher than that in the C5a+C5aRA group (*P* < 0.05), as shown in Figure 7.

## 4. Discussion

The complement system is a significant component of innate immunity, composed of more than 30 kinds of complement proteins, and widely exists in the body [10]. Anaphylatoxin C5a is a complement peptide chain fragment released by the complement system during the activation process. It is composed of 74 amino acid residues and is a kind of inflammation-promoting protein. In injured brain tissue, C5a may be involved in the functional regulation of neurons and glia [11]. C5a mainly binds to specific G protein-coupled receptors on the cell membrane's surface and exerts anaphylactic toxic effects. Microglia, astrocytes, and neurons in the central nervous system can secrete complement C5a under abnormal stimulation C5a [12, 13]. Research suggests that C5a can activate microglia and promote the secretion of proinflammatory cytokines and harmful substances such as oxygen free radicals and NO. It can also assemble around the inflammation areas by attracting some neutrophils and phagocytes with specific receptors, thus further amplifying the local inflammatory response [14]. The C5a-mediated inflammatory response may cause secondary inflammatory damage to tissues. Also, the C5a-mediated inflammatory response can form a neurotoxic inflammatory environment in tissues, resulting in neuronal dysfunction. Hence, it was involved in inflammatory demyelinating lesions and other inflammation-related central neuropathy [15].

Specific binding of C5a/C5aR is an important way to induce the complement cascade reaction and to promote the development of inflammation. Nevertheless, the study revealed that C5a employs a neuroprotective effect against glutamate-mediated neurotoxicity [16, 17]. The NMO models were constructed in WT mice and C5aR-/- mice to investigate the role of C5a and its receptor C5aR in NMO. In an *in vitro* model, the effects of C5a and its receptor C5aR on Glu concentration and NMDAR protein expression levels during the pathogenesis of NMO were preliminarily explored from the levels of spinal cord tissue and optic nerve tissue. AQP4 is a class of water channel transmembrane protein expressed on the foot processes of astrocytes, which plays a vital role in maintaining the water balance of brain parenchyma, extracellular osmotic pressure, promoting glial cell migration, and changing neuronal activity [18, 19]. GFAP is a skeleton protein of astrocytes in the central nervous system playing a crucial conditioning role in the complement-mediated spinal cord and optic nerve injury [20, 21]. First, an immunofluorescence assay was used to detect the expression of AQP4 and GFAP in spinal cord tissue and optic nerve tissue, respectively, and spinal cord injury in an *in vitro* model was rated (with scores). The experimental result showed no AQP4 and GFAP staining loss was observed in the control group's spinal cord and optic nerve tissue. In the WT, C5aR-/-, C5a, and C5a+C5aRA groups, AQP4 and GFAP staining loss was observed to varying degrees. Compared with the control group, the ASIA motor score of the WT, C5aR-/-, C5a, and C5a+C5aRA groups was significantly higher, the ASIA motor score of the C5aR-/- group was significantly higher than that of the WT group, and the loss rate of AQP4 and GFAP staining in the C5aR-/- group was also significantly higher than that in the WT group. Hence, it is suggested that NMO can cause the deletion of AQP4 and GFAP in the spinal cord and optic nerve tissue, and the deletion of C5aR is related to the deletion of AQP4 and GFAP in the NMO model to some degree. For the sake of identifying the relationship between the deletion of C5aR and the deletion of AQP4 and GFAP in the NMO model, human recombinant C5a intervention and human recombinant C5a+C5aR inhibitor intervention were performed in the WT mice models. The experimental result showed that the ASIA motor score in the C5a+C5aRA group was significantly higher than that in the C5a group. The proportion of AQP4 and GFAP staining deletion was also significantly higher than that of the C5a group, suggesting that the loss rate of C5aR may participate in the regulation of the expression of AQP4 and GFAP in the NMO model and show a certain promoting effect on the deletion of AQP4 and GFAP.

Glutamate is a crucial excitatory neurotransmitter in the central nervous system. It can activate the ionic glutamate receptor (NMDAR) by mediating the uptake and/or transport barrier and inducing oligodendrocytes' toxic excitatory injury. Thus, it can induce demyelination in the central nervous system and optic nerve [22]. Research showed that glutamate and its receptors showed significantly higher in acute myelin injury sites in multiple sclerosis patients. NMDAR, a highly selective inhibitor, can improve nerve defects and inflammatory response of spinal cord tissue in animal models of multiple sclerosis. It also alleviates myelin sheath and axon loss [23, 24]. This infers that Glu and receptors may play a role in the pathogenesis of NMO. Besides, the expressions of NMDAR1 and NMDAR2B in spinal cord tissue and optic nerve tissue samples of each group were detected.

At the same time, the concentration of Glu in the culture solution of each sample was detected. Results showed that, compared with the control group, the protein levels and Glu concentrations of NMDAR1 and NMDAR2B in the spinal cord and optic nerve tissues of the WT, C5aR-/-, C5a, and C5a+C5aRA groups were significantly higher. The protein levels and Glu concentration of NMDAR1 and NMDAR2B in the C5aR-/- group were significantly higher than those in the WT group, and the protein expression levels and Glu concentration of NMDAR1 and NMDAR2B in the C5a+C5aRA group were significantly higher than those in the C5a group. It indicated that C5a and its receptor could regulate glutamate concentration by regulating NMDAR activity in spinal cord tissue and optic nerve tissue, which affects the occurrence of NMO. In this regard, the regulatory effect of C5a on the loss of AQP4 and GFAP in NMO that was mentioned before was confirmed again. In this study, the effect of C5a receptor deletion on NMDAR activity and neurotoxicity of Glu has not yet been made apparent. Thus, future studies will further strengthen the role of C5a- and C5aR-related signaling pathways.

Taken together, in the NMO model, C5a receptor deletion induces increased NMDAR expression in spinal cord and optic nerve tissue, which promoted the excitotoxic effect of glutamate. In response to this, the deficiency of AQP4 and GFAP aggravates and the course of NMO was further aggravated.

## Figures and Tables

**Figure 1:** Comparison of ASIA motor scores in each group. ^∗^*P* < 0.05.

**Figure 2:** Comparison of the expression of AQP4 and GFAP in spinal cord tissue samples of each group.

**Figure 3:** Comparison of the expression of AQP4 and GFAP in optic nerve tissue samples of each group.

**Figure 4:** Comparison of protein expressions of spinal cord tissue samples in NMDAR1 and NMDAR2B in each group. ^∗^*P* < 0.05 and ^∗∗^*P* < 0.01.

**Figure 5:** Comparison of the protein expression of NMDAR1 and NMDAR2B in optic nerve tissue samples of each group. ^∗^*P* < 0.05 and ^∗∗^*P* < 0.01.

**Figure 6:** Comparison of Glu concentration in culture solution of spinal cord tissue of each group.

**Figure 7:** Comparison of Glu concentration in culture solution of optic nerve tissue of each group. ^∗^*P* < 0.05 and ^∗∗^*P* < 0.01.

## Data Availability

The datasets during the current study are available from the corresponding author on reasonable request.
